The article "Analysis and early warning management of resource and environmental carrying capacity in agricultural provinces: A case study of Henan Province" was retracted in 2025. Reasons: unreliable results or conclusions; concerns about the peer review; concerns about the authorship.

# Analysis and early warning management of resource and environmental carrying capacity in agricultural provinces: A case study of Henan Province

**DOI:** 10.1371/journal.pone.0318848

**Published:** 2025-02-12

**Authors:** Weidong Chen, Meng Lian

**Affiliations:** Tianjin University School of Economics and Management, Tianjin, China; China West University, CHINA

## Abstract

Resources and Environmental Carrying Capacity (RECC) is a comprehensive concept that encompasses the interactions between resources, the environment, and human activities, serving as the foundation for social development strategies. To adequately reflect this complex relationship, a multi-level, multi-dimensional evaluation indicator system must be developed. This paper constructs a regional soil environmental evaluation system incorporating PM2.5 indicators, which is in line with relevant environmental protection policies and planning orientations in our country from 2014 to 2023. It analyzes the level and development trend of RECC in Henan Province and proposes measures for effective management. The results indicate the following: (1) The RECC in Henan Province demonstrates a downward trajectory, marked by temporary fluctuations over time. It hit its nadir in 2019, subsequently undergoing a gradual resurgence; (2) Analysis of individual dimension indicators reveals that the natural carrying capacity has declined from a medium to a relatively weaker level. Meanwhile, environmental carrying capacity has shown a slight downward trend but has generally remained stable. In contrast, socio-economic carrying capacity has demonstrated an upward trend, rising from a medium to a relatively strong level. In terms of early warning measures, it is essential to establish a red warning zone, implement a credit record accountability system, and develop a monitoring warning database along with an information technology platform. This paper demonstrates that the indicator system is effective for evaluating RECC across different dimensions and holds significant reference value for assessing RECC in similar regions.

## 1. Introduction

Resources and the environment form the foundation for human survival. Since the 20th century, advancements in technology have significantly boosted social productivity and civilization. However, limited understanding of the relationship between resource use and sustainable development has led to overconsumption, pollution, and intensified conflicts between environmental health and economic growth [1]. Economic expansion following reforms further exposed the limitations of traditional, extensive growth models, creating resource bottlenecks and environmental capacity constraints [2, 3]. For example, uneven water distribution and pollution have exacerbated shortages, particularly in arid regions, disrupting agriculture, industry, and daily life [4]. Similarly, urbanization and industrialization have increased wastewater, exhaust gas, and waste residue emissions, causing severe environmental issues [5, 6].

To address these challenges, Masijun introduced the concept of a "society-economy-nature" composite ecosystem, emphasizing the interdependence of humans and nature. This framework integrates societal, economic, and environmental subsystems and serves as a foundation for sustainable development [7]. The core of this framework is RECC, indicating a region’s capacity to support social and economic activities without harming environmental stability [8–12]. RECC integrates ecological, social, and economic dimensions, setting thresholds for human activity to ensure resilience and long-term development [13–19].

Urbanization has heightened RECC-related challenges, including population pressure, resource overuse, and pollution, leading to urban systems exceeding their adaptive capacity [7]. In response, China’s ecological civilization reforms have introduced monitoring and early warning mechanisms for RECC to support sustainable growth. Originally rooted in ecology, the concept of carrying capacity has evolved to encompass broader dimensions of development, including resource management, urban planning, and disaster resilience [20–27].

Evaluation methods for RECC include ecological footprint analysis, energy analysis, system dynamics, and comprehensive indicator-based approaches [28–40]. While these methods provide insights, they often lack regional specificity, neglect interactions among resources, and over-rely on generalized indicators, limiting their applicability [41–43]. This study builds on existing research by constructing a regional soil environmental evaluation system incorporating PM2.5 indicators. By addressing interactions between soil and atmospheric environments, this system offers a novel approach for assessing and managing regional environmental quality, aligned with China’s environmental policies from 2014 to 2023.

## 2. Methods and methods

### 2.1. Research area characteristics

Henan Province, situated in the central and eastern region of China along the middle and lower reaches of the Yellow River, boasts fertile land and a favorable climate ideal for crop cultivation. Historically, it has been a key agricultural hub in China. These natural advantages position Henan as a leader in agricultural development.

As one of the country’s major agricultural provinces, Henan ranks among the top three nationwide in agricultural output, contributing over 8.5% of the national crop planting area, consistently exceeding 220 million acres. The province excels in grain production, with wheat and corn holding significant national prominence. Other crops, such as oilseeds, vegetables, and fruits, have also seen steady growth. Notable outputs include: Peanuts: Nearly 90% of the national total. 2. Vegetables: Over 76 million tons annually. 3. Fruits: Approximately 25 million tons annually.

Animal husbandry in Henan has also developed steadily, with pork and poultry production driving increases in meat output. The province slaughters nearly 60 million pigs annually, with poultry egg production exceeding 4.5 million tons, and milk output showing consistent growth for four years. Henan’s agricultural development is further supported by technological advancements, such as the introduction of the Kainong 1 high oleic acid peanut variety and the Henan Agricultural Machinery Cloud Platform, which have infused new vitality into the sector [44–48].

### 2.2 Methodology

The Analytic Hierarchy Process (AHP) is a system analysis method that combines qualitative and quantitative analysis, proposed by the famous American operations research expert Professor T.L. Saaty in the 1970s. This method is mainly used to deal with complex decision-making problems. By breaking down a complex-making problem into multiple levels, each level containing several criteria or alternatives, it helps decision-makers to better understand the problem and make the optimal decision [49, 50].

The Analytic Hierarchy Process (AHP) initially breaks down complex decision-making problems into multiple sub-problems or factors, forming a structure. This decomposition aids in simplifying the problem, allowing decision-makers to clearly visualize the various components of the problem. By constructing a hierarchy, AHP incorporates sub-problems or factors into a unified system for consideration. This helps decision-makers to comprehensively and systematically evaluate all relevant factors, avoiding partial or localized decisions. At each level of the hierarchy in AHP, decision-makers need to compare each factor or criterion pairwise to determine their relative importance. This comparison helps to reveal the priority relationships between different factors. The main steps of AHP involve breaking down the complex decision-making problem into multiple levels, conducting pairwise comparisons of the elements at each level calculating the relative importance weights of each element, and finally integrating these weights to select the optimal solution. This method is particularly effective in dealing with complex multi-factor decision problems, helping decision-makers to systematically analyze and solve problems [22].

### 2.3 Constructing an evaluation indicator system

RECC is influenced by various factors, therefore, it is necessary to construct a multi-level, multi-objective indicator evaluation system. When developing the evaluation indicator system, all these factors must be considered to ensure that the system can fully reflect the multi-dimensional characteristics of RECC. For instance, resource consumption, environmental impact, and socio-economic conditions can be used as first-level indicators, which can be further refined into second-level indicators such as energy consumption, pollutant emissions, and per capita GDP [51, 52]. This hierarchical refinement allows for a more precise quantification and evaluation of various aspects of RECC, providing a basis for decision-makers. Additionally, the construction of the evaluation indicator system should also consider the interactions and influences between indicators, as well as their overall impact on RE, to ensure the accuracy and practicality of the evaluation results. This paper follows the principles of scientificity and feasibility, selecting 17 specific indicators to the evaluation system (Table **1**), then divides them into three dimensions according to different regions, namely the target layer (A), the criterion layer (B), the scheme layer (C).

**Table 1:** Indicator evaluation system table.

Target layer	Criteria Level	Solution Level	Specific indicators	unit	direction
	Carrying capacity of natural resources(B1)	Land resources(C1)	Per capita arable land area(D1)	hectare/person	+
			Per capita construction land area(D2)	m^2^/person	+
		Water resources(C2)	Per capita water resources(D3)	m^3^/person	+
			Per capita water consumption(D4)	m^3^	+
		Energy resources (C3)	Total energy consumption(D5)	ten thousand tons of standard coal	-
RECC(A)			Energy consumption per GDP(D6)	tonnes of standard coal per million yuan	-
		Forest resources(C4)	Forest coverage rate(D7)	%	+
			Afforestation area(D8)	million hectares	+
	Environmental carrying capacity(B2)	Water environment (C5)	Chemical Oxygen Demand Emissions (D9)	Ten thousand tons	-
			Ammonia nitrogen emission(D10)	Ten thousand tons	-
		air environment(C6)	Sulfur dioxide emission(D11)	Ten thousand tons	-
			Nitrogen oxides (D12)	Ten thousand tons	-
			Particulate Matter (PM2.5)(D13)	Ten thousand tons	-
	socio-economic carrying capacity (B3)	Level of social development(C7)	Per capita GDP (D14)	yuan/person	+
			Urbanization rate(D15)	%	+
		Level of social development(C8)	Contribution rate of the primary industry(D16)	%	+
			Industrial contribution rate(D17)	%	+

#### 2.3.1 Data processing

This paper employs the range standardization method from standardized methods to process the data. Data standardization is the process of transforming raw data through certain mathematical into dimensionless and magnitude-free standardized values. After processing, the data, regardless of whether the original values are positive or negative, satisfy 0≤X≤1, and both positive and negative indicators can be transformed into positive indicators. This processing aims to eliminate differences brought by characteristics such as the nature, dimension, and magnitude different variables, so that the values of each indicator are at the same magnitude level, thus facilitating comprehensive analysis and comparison.

Normalize the factors based on the number of options for each. Since the platform includes both "positive indicators" and "negative indicators," these two types of data will be preprocessed separately. Here, to accommodate the situation where an entire column has the same value, we subtract 0.0001 from the minimum value and add 0.0001 to the maximum value. This adjustment has a negligible impact on the overall results and can therefore be ignored.


$$\begin{array}{l} X_{\min}=\min(X_{1j},X_{2j},\cdots X_{nj})-0.001\\ X_{\max}=\max(X_{1j},X_{2j},\cdots X_{nj})+0.001 \end{array}$$

Processing of positive indicators:

$$Z_{ij}=\frac{X_{ij}-X_{\min}}{X_{\max}-X_{\min}}$$ (1)

Processing of negative indicators:

$$Z_{ij}=\frac{X_{\max}-X_{ij}}{X_{\max}-X_{\min}}$$ (2)

In this context, X_ij_ represents the normalized data. By calculating the scores for each influencing factor, we can determine the ranking of all factors’ importance Table **2** shows the standardized results of the evaluation indicators.

**Table 2:** Standardized indicator values.

	2014	2015	2016	2017	2018	2019	2020	2021	2022	2023
D1	1.0000	0.9311	0.8625	0.8153	0.8350	0.0641	0.0000	0.0858	0.1132	0.2148
D2	0.0000	0.8183	0.9193	0.9726	0.9974	1.0000	0.8940	0.8704	0.7266	0.4553
D3	0.2343	0.2387	0.3312	0.4936	0.3305	0.0000	0.4568	1.0000	0.1561	0.5898
D4	0.2857	0.6714	0.7800	0.9371	0.9343	1.0000	0.7686	0.3657	0.5343	0.0000
D5	0.3114	0.0774	0.0689	0.0000	0.2126	0.0590	0.2524	0.5727	0.9448	1.0000
D6	1.0000	0.7751	0.5943	0.3669	0.2133	0.0674	0.0833	0.0280	0.0000	0.0644
D7	0.0000	0.1198	0.6587	0.8982	0.4431	0.1317	1.0000	0.4192	0.4193	1.0000
D8	1.0000	0.5565	0.0650	0.2602	0.3617	0.5307	0.6393	0.4109	0.1168	0.0000
D9	0.6180	0.5957	0.0230	0.0000	0.0557	0.6994	0.7063	0.7571	0.9861	1.0000
D10	1.0000	0.9478	0.2268	0.1954	0.1223	0.0282	0.1014	0.0000	0.0345	0.1745
D11	1.0000	0.9526	0.3117	0.1994	0.1546	0.0923	0.0071	0.0010	0.0000	0.0018
D12	1.0000	0.8339	0.3624	0.2118	0.1443	0.5659	0.0903	0.0405	0.0000	0.3821
D13	1.0000	0.9557	0.4421	0.1884	0.1736	0.3818	0.0197	0.0037	0.0000	0.0259
D14	0.0000	0.0902	0.2046	0.3729	0.5639	0.7033	0.7162	0.8653	1.0000	0.9232
D15	0.0000	0.1512	0.2863	0.4229	0.5518	0.6876	0.7966	0.8749	0.9225	1.0000
D16	0.1183	0.1479	0.1361	0.1420	0.0710	0.0000	1.0000	0.4260	0.7041	0.3432
D17	1.0000	0.8405	0.6769	0.6933	0.6994	0.7832	0.0000	0.3211	0.8896	0.5849

### 2.4 Establishment and calculation of AHP weights

The fundamental principle of AHP is based on the nature of the problem and the objectives, it requires experts to quantitatively evaluate the relative importance factors at each level according to the inter-factor interactions and the membership relationships of the hierarchical clustering, and to determine the weight order, and then calculate the combined weights relative importance. In this study, based on expert experience, the relative importance of two indicators at adjacent levels in the evaluation indicator system was determined. to the scoring results, the indicators at the same level were compared in pairs, and three decision-making matrices (Table 3) were constructed and calculated to determine relative importance of B1, B2, and B3 indicators through the comparison pairs.

**Table 3:** RECC decision matrix.

A	B1	B2	B3
B1	1	1/3	1/5
B2	3	1	1/3
B3	5	3	1
*λ* max = 3.039, CI = 0.019, CR = 0.037			

The computation results of the Analytic Hierarchy Process show that the maximum eigenvalue is 3.039. According to the RI table, the corresponding RI value is 0.525. Therefore, CR = CI/RI = 0.037<0.1, passing the consistency test. The weight results of all indicators are shown in Table **4**.

**Table 4:** RECC indicator weights.

Target layer	Criterion layer	weight value	Solution layer	weight value	Specific indicators	weight value
A	B1	0.4395	C1	0.1283	D1	0.0981
					D2	0.0302
			C2	0.1007	D3	0.0597
					D4	0.0410
			C3	0.1137	D5	0.0615
					D6	0.0522
			C4	0.0968	D7	0.0477
					D8	0.0491
	B2	0.3456	C5	0.0966	D9	0.0445
					D10	0.0521
			C6	0.2490	D11	0.0685
					D12	0.0735
					D13	0.1070
	B3	0.2149	C7	0.0860	D14	0.0339
					D15	0.0521
			C8	0.1289	D16	0.0424
					D17	0.0865

### 2.5 Comprehensive evaluation of RECC

Based on the standardized results of the entropy method (Table **1**) and the AHP weight results (Table **4**), the comprehensive evaluation results of RE are as follows (Table 5):

**Table 5:** RECC evaluation results.

	2014	2015	2016	2017	2018	2019	2020	2021	2022	2023
D1	0.0981	0.0913	0.0846	0.0800	0.0819	0.0063	0.0000	0.0084	0.0111	0.0211
D2	0.0000	0.0247	0.0278	0.0294	0.0301	0.0302	0.0270	0.0263	0.0219	0.0138
D3	0.0140	0.0142	0.0198	0.0295	0.0197	0.0000	0.0273	0.0597	0.0093	0.0352
D4	0.0117	0.0275	0.0320	0.0384	0.0383	0.0410	0.0315	0.0150	0.0219	0.0000
D5	0.0521	0.0496	0.0162	0.0104	0.0081	0.0048	0.0004	0.0001	0.0000	0.0001
D6	0.0424	0.0354	0.0154	0.0090	0.0061	0.0240	0.0038	0.0017	0.0000	0.0162
D7	0.0213	0.0053	0.0047	0.0000	0.0146	0.0040	0.0173	0.0392	0.0647	0.0685
D8	0.0735	0.0570	0.0437	0.0270	0.0157	0.0050	0.0061	0.0021	0.0000	0.0047
D9	0.0865	0.0827	0.0382	0.0163	0.0150	0.0330	0.0017	0.0003	0.0000	0.0022
D10	0.0000	0.0043	0.0098	0.0178	0.0269	0.0335	0.0342	0.0413	0.0477	0.0440
D11	0.0000	0.0074	0.0141	0.0208	0.0271	0.0338	0.0391	0.0430	0.0453	0.0491
D12	0.0053	0.0066	0.0061	0.0063	0.0032	0.0000	0.0445	0.0190	0.0313	0.0153
D13	0.0521	0.0438	0.0353	0.0361	0.0364	0.0408	0.0000	0.0167	0.0463	0.0305
D14	0.0000	0.0074	0.0405	0.0552	0.0273	0.0081	0.0615	0.0258	0.0258	0.0615
D15	0.0522	0.0291	0.0034	0.0136	0.0189	0.0277	0.0334	0.0215	0.0061	0.0000
D16	0.0661	0.0637	0.0025	0.0000	0.0060	0.0748	0.0756	0.0810	0.1055	0.1070
D17	0.0339	0.0321	0.0077	0.0066	0.0041	0.0010	0.0034	0.0000	0.0012	0.0059

According to the comprehensive score values in the above table, we can use Formula (3) to calculate the final results of the target layer, criterion, and scheme layer.


$$A=\sum_{i=1}^{n}\left(W_{i}\times B_{i}\right)$$ (3)

## 3. Results

Over the past decade, the RECC in Henan Province has shown a significant downward trend, transitioning from a moderate level to a weaker one. In terms of natural resources and environmental carrying capacity, Henan Province has experienced a dual decline. The carrying capacity of natural resources has decreased from a moderate level to a weaker state, which is related to factors such as the tension of land resources caused by urban expansion, the over-exploitation of water resources, and the unreasonable exploitation of mineral resources. More seriously, the environmental carrying capacity has significantly decreased from a relatively strong state to a weaker level, with a decline that cannot be ignored. This change directly points to the severe challenges faced by Henan Province in terms of air quality, water body quality, soil health, and ecosystem stability. Issues such as the increase in industrial emissions, the intensification of the urban heat island effect, and the reduction of green space have all exerted tremendous pressure on the environmental carrying capacity. Although during this period, the socio-economic carrying capacity of Henan Province has been enhanced, slightly improving from a weaker baseline, it is still relatively weak, indicating that the contradiction between economic development and resource and environmental support remains prominent. See Table 6 for details

**Table 6:** RECC score for Henan Province.

	2014	2015	2016	2017	2018	2019	2020	2021	2022	2023
C1	0.0981	0.1160	0.1124	0.1094	0.1120	0.0365	0.027	0.0347	0.0330	0.0394
C2	0.0257	0.0417	0.0518	0.0679	0.0580	0.0410	0.0588	0.0747	0.0312	0.0352
C3	0.0945	0.085	0.0316	0.0194	0.0142	0.0288	0.0042	0.0018	0.0000	0.0163
C4	0.0948	0.0623	0.0484	0.027	0.0303	0.009	0.0234	0.0413	0.0647	0.0732
C5	0.0865	0.087	0.048	0.0341	0.0419	0.0665	0.0359	0.0416	0.0477	0.0462
C6	0.0574	0.0578	0.0555	0.0632	0.0667	0.0746	0.0836	0.0787	0.1229	0.0949
C7	0.0522	0.0365	0.0439	0.0688	0.0462	0.0358	0.0949	0.0473	0.0319	0.0615
C8	0.1000	0.0958	0.0102	0.0066	0.0101	0.0758	0.0790	0.0810	0.1067	0.1129
B1	0.3131	0.3050	0.2442	0.2237	0.2145	0.1153	0.1134	0.1525	0.1289	0.1641
B2	0.1439	0.1448	0.1035	0.0973	0.1086	0.1411	0.1195	0.1203	0.1706	0.1411
B3	0.1522	0.1323	0.0541	0.0754	0.0563	0.1116	0.1739	0.1283	0.1386	0.1744
A	0.6092	0.5821	0.4018	0.3964	0.3794	0.3680	0.4068	0.4011	0.4381	0.4796

Table 6 shows the dimensions and specific indicator scores of RECC in Henan Province. First, let’s look at the target level (A) From 2014 to 2023, the overall RECC in Henan Province decreased from 0.6092 in 2014 to 0.4796, a decrease of 21.3%. This trend is characterized by fluctuations, reaching the lowest point in 2019, and then gradually recovering. The main reason for this is the imbalance in the development between the resource layer and the economic and environmental layers from 2014 to 2018. In other words, the development of the environment and economy lagged behind the development of natural resources, leading to a lack of coordinated development among resources, environment, and economy.

From the perspective of the criterion layer, the carrying of natural resources has gradually decreased. with an overall of 46.7%. In terms of land resources, the per capita arable land area continues to decline while the per capita construction land continues to increase. The continuous increase in construction land has led to a mismatch in land resources, affecting the carrying capacity of land resources. The overall trend of water resources carrying capacity is stable, without significant fluctuations. The carrying capacity of energy and forest resources both show an upward trend, especially energy, which has increased by nearly 83%.This indicates that the Henan Province has made certain achievements in energy consumption and greening during this period.

Environmental carrying capacity (B2) was the lowest in the three years from 2016 to 2018. The main reason is the unrestricted discharge of wastewater and the lack of environmental awareness, which leads to pollutants in the water that cannot be diluted. Additionally, industrial gas emissions and numerous construction projects without dust prevention measures have caused sulfur dioxide and PM2.5 levels in the air to severely exceed standards. PM2.5, due to its small particle size, can directly enter the alveoli of the human body, deposit in the lungs, and even enter other organs through the circulatory system. In addition, PM2.5 may also become a carrier for bacteria and viruses, promoting the transmission of respiratory infectious diseases. At the same time, PM2.5 may also settle in the soil and water bodies, causing pollution to the soil and water quality, and further affecting the stability of the ecosystem. After 2018,continuously promote returning farmland to forest and grass, the Green Mountain Project, etc., and strengthen the protection and restoration of forest, wetland, grass and other ecosystems. Strictly implement the ecological protection red line system, and strictly protect important ecological function areas. under the background of green development, water and air environments have been effectively controlled and gradually recovered.

The economic carrying capacity (B3) plummeted sharply between 2016 and 2018, primarily due to the industry’s dominance in GDP contribution, which led to a severe mismatch between industry and the first sector during this period. The social development of Henan Province has been influenced by demographic factors, with a rapid shift of the population towards urban areas over the past decade. This could be one of the main reasons for the significant changes the province’s socio-economic carrying capacity. With the acceleration of urbanization, for example, Xuchang City has set up a high-level urbanization work and urban-rural integrated development work group led by the Party Secretary and mayor, and has started to compile a number of supporting policies, forming a policy system of "1 6 16", the urban-rural structure of Henan Province has undergone profound changes, with a large number of rural residents flooding into cities in search of more job opportunities and better living conditions. This population movement has not only altered the demographic distribution of Henan Province, but has also put higher demands on urban infrastructure, educational resources, and healthcare. In the process of urbanization, the economic structure and social organization of Henan have been continuously adjusted and optimized to meet the challenges brought by population growth. Therefore, the rapid urbanization of the population is not only a social phenomenon but also an important factor influencing the socio-economic development of Henan Province.

In order to better understand the weight values of Henan Province’s resource and environmental carrying capacity, we divide the weight index into four levels: weak relatively weak, general, and relatively strong. See Table **7** for the specific classification of carrying capacity levels.

**Table 7:** Load capacity rating.

level	Resource and environmental carrying capacity (0,1)	Natural resource carrying capacity(0,0.4395)	Environmental carrying capacity(0,0.3456)	Socio-economic carrying capacity (0,0.2149)
weak	(0, 0.25)	(0, 0.1099)	(0, 0.0864)	(0, 0.0537)
relatively weak	(0.25, 0.5)	(0.1099, 0.2198)	(0.0864, 0.1728)	(0.0537, 0.1074)
medium	(0.5, 0.75)	(0.2198, 0.3296)	(0.1728, 0.2592)	(0.1074, 0.1611)
strong	(0.75, 1)	(0.3296, 0.4395)	(0.2592, 0.3456)	(0.1611, 0.2149)

As can be seen from Table 7, within the time span from 2014 to 2023, the natural resource capacity of Henan Province has undergone significant changes, decreasing from a moderate level to a relatively weaker level. Meanwhile, although the environmental carrying capacity has shown a slight trend, it has overall remained at a relatively weak level. Notably, during this period, the socio-economic carrying capacity has shown a positive upward trend, rising a moderate level to a relatively strong level.

## 4. Early warning management

The changes in Henan Province’s resource and environmental carrying capacity, especially those that are relatively weak or declining, have created an urgent need for early management. We recommend:

### 4.1 Comprehensive supporting measures

Implement the strictest regional restrictions based on overloading factors Legally suspend the approval procedures for new, renovated, and expanded projects in related industries, and specify the timeline for the exit of industries causing the overload. When enterprises, institutions and other producers and operators exceed the pollutant emission standards or exceed the total control indicators for the emission of key pollutants, environmental protection departments of the people’s governments at or above the county level may order them to take measures such as restricting production and suspending production for rectification. If polluter discharges pollutants through concealed pipes, soakage wells, soakage pits, injection or by tampering with and forging monitoring data, or by not operating pollution facilities normally, and exceeds the pollutant emission standards, the environmental protection department may also order it to take measures such as suspending production for rectification. Meanwhile, implement a reduction in urban construction land and legally penalize enterprises that severely damage resource and environmental carrying capacity and violate laws by polluting and destroying ecological resources near overloaded areas. Handle these cases according to the single-item control measures for the overloaded areas, such as those related to water resources, land resources, the environment, ecology, and the sea. Implement reward measures of different degrees for areas that have transformed from overload to near overload or from near overload to non-overload. Establish a credit record for governments and enterprises that fail to implement restrictive measures or continue to deteriorate resource and environmental conditions, and include them in the information sharing platform. Pursue legal and regulatory responsibilities strictly.

### 4.2 Water resources management measures

1. Suspend the approval of new water withdrawal permits for construction projects, formulate and implement a water use reduction plan, apply stricter water-saving standards in key water use sectors, reduce unreasonable irrigation areas, implement a differentiated water resources fee policy, and promote pilot reforms of the water resources tax.

2. Suspend the approval of high water-consuming projects, strictly control the total water, increase efforts in water saving and utilization of unconventional water sources, and optimize industrial structure adjustment.

3. Strictly control the total resources consumption and intensity, strengthen water resources protection and river pollution control.

### 4.3 Land resource management measures

1. Implementing Farmland Compensation Balance: When construction projects occupy farmland, principle of "occupy as much, reclaim as much" must be followed. This ensures that the total amount of farmland does not decrease by reclaiming far that is equivalent in both quantity and quality to the occupied farmland.

2. Improving Farmland Quality: Enhancing farmland quality through soil improvement, construction agricultural water conservancy facilities, and other measures to increase grain production capacity.

3. Construction Land Management: Strictly enforcing construction land standards: When construction projects need use land, they must comply with the national spatial planning, annual land use plan, and land use control requirements, and strictly adhere to the construction land standards.

Promoting Economical and Intensive Land Use: Encouraging the adoption of multi-story buildings, underground space development, and other methods to save land and enhance the efficiency of construction land use.

### 4.4 Ecological management measures

1. Develop a time-limited ecological restoration plan, implement stricter regular precision systems, and if necessary, carry out ecological immigration relocation. Enforce a closure management system in areas with severely degraded ecosystems to promote natural ecological recovery.

2. Intensify monitoring of areas at risk of ecological function degradation. Scientifically implement restoration and management of mountains, rivers, forests, farmland and lakes. Reasonably disperse the population to curb the trend of ecosystem degradation.

3. Establish a mechanism for realizing the value ecological products. Utilize investment, fiscal, and financial policy tools to support the development of green and ecological economy.

### 4.5 Construction of monitoring and warning database information technology platform

1. Establish a multi-departmental collaborative layout mechanism for monitoring stations, focusing on strengthening weak links and the establishment of county monitoring points. Achieve full coverage of the national resource and environmental carrying capacity monitoring network.

2. Integrate and compile monitoring data from various departments resource and environmental carrying capacity. Construct a monitoring and warning database, utilizing cloud computing, big data processing, and data fusion technology to achieve real-time data sharing dynamic updates.

## 5. Discussion

Limitations of this study: Firstly, the core purpose of the AHP method is to identify the optimal plan among multiple plans, but it does not have the ability to propose innovative methods to solve problems, so it has shortcomings in terms of innovation. Secondly, when AHP is used to analyze multiple indicators or dimensions that influence each other, it is necessary to construct a multi-level, large-scale judgment matrix. However, due to the complex interaction relationship between indicators, the difficulty of analysis increases with the increase in the number of indicators. Finally, there may be problems in the rationality of the judgment matrix constructed in this study. This is because the matrix is constructed on the basis of subjective scoring by experts, and subjective scoring often has a certain degree of subjectivity and bias. Therefore, it may be affected by these biases when calculating the weights, which in turn reduces the recognition and credibility of the analysis conclusion.

So far, research results of RECC are abundant. However, affected by regions and scales, the interaction relationship between resources, environment, and economy becomes very complex. Meanwhile, the cross-scale issues in China’s eastern, southern, western, northern, and central regions lead to difficulties in RECC research., in the era of big data and the rise of various supporting software (GIS), we should strengthen the construction and development of simulation models related to RECC and support tools for RECC analysis.

## 6. Conclusion

The evaluation of RECC is a complex process encompassing resources, environment, and economy. This study integrates the PM2.5 indicator into the AHP-based evaluation system, refining the assessment framework. Results reveal Henan Province faces challenges in natural resource utilization and sustainable development, requiring enhanced resource management and green initiatives. Economic carrying capacity can improve through strategies like optimizing industrial layouts and urban planning. The study demonstrates the value of a differentiated index system for accurately reflecting regional conditions, providing insights for policy formulation. These findings not only align with Henan’s situation but also offer guidance for similar regions addressing sustainability challenges.
